# Analysis of Ice and Snow Path Planning System Based on MNN Algorithm

**DOI:** 10.1155/2022/1586006

**Published:** 2022-03-07

**Authors:** YinZhe Jin, Bai Li

**Affiliations:** ^1^Post-Doctoral Research Center of Skiing Teaching and Training Base, Harbin Sport University, Harbin, Heilongjiang, China; ^2^School of Sports Science, Lingnan Normal University, Zhanjiang, Guangdong, China; ^3^School of Kinesiology and Health Promotion, Dalian University of Technology, Dalian, Liaoning, China

## Abstract

Traditional ice and snow path planning methods still have internal environmental problems in intelligent path planning, such as weak innovation ability, imperfect management, long planning path, unreasonable security structure, and low degree of specialization. Therefore, more and more ice and snow sports lovers are eager to solve this problem. This paper designs a path planning method based on three-dimensional ice and snow model. The path planning method of moving snow and ice based on MNN (Multiclass Neural Networks) algorithm is studied from many aspects. MNN algorithm is used for comprehensive analysis and evaluation. The mobile phone provides data information on key nodes, air resistance, momentum change, ice and snow movement track, and so on. The results show that the ice and snow path planning system based on MNN algorithm designed in this paper has the advantages of high feasibility, high data accuracy, and good prediction effect and can effectively improve the efficiency of ice and snow path planning.

## 1. Introduction

According to the survey, the research on ice and snow movement track in sports mainly focuses on the movement type, path planning method, and optimal movement strategy and rarely constructs the change law of movement path process and intelligent algorithm [1]. On the other hand, some foreign scholars have begun to reconstruct the track of ice and snow in sports, which is used to analyze the tactical strategy between teams in sports, and have verified the effectiveness of the track of ice and snow through experiments [2]. At present, the existing sports path planning model provides a lot of reconstruction methods, but there are few targeted breakthroughs in ice and snow sports [3]. In this context, this paper proposes a path planning model of sports ice and snow based on MNN algorithm.

The innovation of this paper lies in the MNN algorithm and ice snow motion path planning algorithm. On this basis, we can make full use of the difference information in the ice and snow movement, carry out multivariate analysis on different types of ice and snow movement data information, combine with MNN algorithm factors, standardize the identification of the path information generated in the process of ice and snow movement, and realize the intelligent planning and correct guidance of ice and snow path according to the characteristics and objectives of ice and snow movement.

This paper studies the construction of intelligent path planning guidance system of ice and snow sports, which is mainly divided into four parts. The first chapter introduces the research background and the general arrangement of this chapter. The second chapter introduces the research status of ice and snow sports and path planning factors. In the third chapter, the dynamic tracking and intelligent path planning model of ice and snow movement based on MNN algorithm is constructed. The Laplace factor method is used to construct the ice and snow movement path planning guidance system and related evaluation system. In Chapter 4, the dynamic tracking and path planning model of ice and snow movement constructed in this paper is verified by experiments, and the conclusion is drawn.

## 2. State of the Art

Since entering the 21st century, there are some problems in the research of ice and snow sports in China, especially in the path planning and intelligent dynamic tracking of ice and snow sports [4]. Based on the sphere kinematics theory and intelligent recognition method, Zenke et al. proposed a method for reconstructing the trajectory of ice and snow movement. According to different types of ice and snow movement rules, they constructed a normalized insurance path planning method [5]. Zhang et al. put forward a unified model of ice and snow movement path based on variational strategy, aiming at the safety and optimal path problems in the process of ice and snow movement, which can solve the problem of multiple dispersion in the process of traditional ice and snow movement [6]. P. Thieberger et al. proposed an antidisturbance optimal planning method for ice and snow sports path based on the types of athletes in ice and snow sports and the low efficiency of cooperation in ice and snow sports [7]. Based on the video tracking strategy, Wang et al. analyzed the path data generated in the process of ice and snow movement according to the genetic algorithm and unified different types of analysis methods. The results were applied to the path planning scheme of ice and snow movement, and the results showed that this method can significantly improve the efficiency of path planning of ice and snow movement [8]. Qi et al. put forward an improved multiangle path optimization analysis model in order to improve the aesthetic effect of athletes in the process of ice and snow sports and obtain the path information of key nodes from common ice and snow sports rules [9]. Bragazzi et al., from the perspective of the planning of the starting point and end point of the path, innovated the determination of the path planning scheme of ice and snow sports and proposed a semiautomatic online path planning method, which can realize remote detection and path planning with the help of cloud computing technology and has certain application value [10]. Fischer et al. scholars analyzed different types of ice and snow movement process from the path planning analysis level and proposed a path optimization analysis method based on ice and snow movement trajectory feedback mode, which can provide the best path planning scheme according to the characteristics of ice and snow movement [11]. In order to reduce the error rate of ice and snow movement in the path planning process, K. W. Guo et al. adopted the multifactor improved strategy docking model and designed verification experiments to verify the stability and reliability of the model in the ice and snow movement path planning process [12]. According to the different types of ice and snow sports, scholars such as Mohammad used different modes of differentiated path analysis methods to classify the types of path planning, then analyzed their differences, and obtained the optimal path scheme according to their shortest distance [13]. Grattarola et al. put forward a path optimization planning model based on firefly tracking algorithm according to the specific ice and snow movement path law, which has the advantages of strong stability and good reliability [14]. According to the characteristics of ice and snow movement path, Miles et al. improved the path planning strategy and proposed an intelligent path planning method based on super-high selection [15]. The research of Janson et al. shows that different types of path optimization strategies can be adopted according to the differences of ice and snow movement; that is, the differences in different path planning schemes can be quickly identified first, and then the common path planning standard schemes can be analyzed point-to-point, and the analysis result data can be converted to the path signal, and the final path planning scheme can be output [16]. Saeed et al. make path planning strategies for different types of ice and snow sports according to their uniqueness. This method can quickly give the shortest path recommendation scheme according to the type of ice and snow sports and the target demand [17].

To sum up, it can be seen that the current ice and snow sports generally have low degree of intelligence, weak applicability, and many restricted conditions in the path planning, which is the same with the study [18, 19]. On the other hand, although there have been many research results in ice and snow sports, there are still many problems in the path planning and guidance of ice and snow sports and few path planning models involving intelligent algorithms [20, 21]. Therefore, it is of great significance to carry out the ice and snow movement path planning method combined with intelligent algorithm.

## 3. Methodology

### 3.1. Application of MNN Algorithm in Intelligent Path Planning of Ice and Snow Sports

At present, genetic algorithm, neural network algorithm, mutual nearest neighbor algorithm, and MNN (multiclass neural network) algorithm are widely used in path planning [21–23]. The so-called mutual nearest neighbor algorithm refers to the process of finding the nearest data in a group of random samples propagating in the state space, replacing the integral operation with the sample mean value, and then obtaining the solution set of the optimal function [24–26]. As long as the global path point contains spatial position information, it can also contain attitude information, which does not need to be related to time, but time information can be considered in local planning. Here, it is specified that the track point is also a kind of path point, that is; when the time constraint is added to the path point information, it can be called a track point. From this point of view, trajectory planning is a kind of path planning. When the path planning process needs to meet the longitudinal and transverse dynamic constraints of ski objects, it becomes trajectory planning. Path planning and trajectory planning can be expressed in both state space and Cartesian coordinate system. In the process of path tracking, the reference path curve can be independent of time parameters. During tracking control, it can be assumed that the unmanned vehicle advances at a constant speed at the current speed, and the driving path approaches the reference path with a certain cost rule. In trajectory tracking, the reference path curve is related to time and space, and the unmanned vehicle is required to reach a preset reference path point within the specified time.

In the research on the optimal solution of the track and path planning of ice and snow sports, in the application process based on MNN algorithm, aiming at the path planning strategy of ice and snow sports, this paper first designs the MNN algorithm based on the influence degree of multidimensional factors. The cloud path location tracking network with strong pertinence is used to formulate the optimal path planning scheme of ice and snow movement and determine the characteristic ice and snow movement trajectory and path planning process. The data processing process of MNN algorithm is shown in Figure 1.

### 3.2. Construction of Intelligent Path Planning Model for Ice and Snow Sports Based on MNN Algorithm

In this model of ice and snow sports path planning based on MNN algorithm, an online guidance scheme based on intelligent path planning strategy is constructed by using three characteristic parameters related to ice and snow sports path and trajectory. Through the research on the track collection, speed control, starting point and end point information, and data analysis strategy in the ice and snow movement, the internal relations of the factors in the whole ice and snow movement path planning guidance system are clearly defined, and the processing process is shown in Figure 2.

The basic steps of building the intelligent path planning model of ice and snow sports can be divided into three steps.

In the first step, we need to find multiple path related optimal detection information with high similarity in morphology and structure from the existing ice and snow motion detection network and then carry out local video tracking to realize the dynamic tracking of the ball in the process of space movement. The tracking function *K*(*s*) is

(1) $$\begin{array}{c} K\left(s\right)=\frac{3s^{3}+3s^{2}+4s+1}{\sqrt{5s+2}}. \end{array}$$

The tracking function *K* ′(*s*) optimized by adding dynamic aggregation factor *t* is

(2) $$\begin{array}{c} K{\;}^{\prime }\left(s\right)=\frac{\sqrt{3s^{3}+3s^{2}+4s+1/\sqrt{5s+2}}}{t+3}, \end{array}$$

where *s* is the track data of ice and snow movement and *t* is the dynamic aggregation factor. In this process, three groups of different types of data are analyzed, and the simulation results are shown in Figure 3. As can be seen from Figure 3, with the increase of data dimension, the tracking function values of different groups of data show a similar change law, and with the increase of data dimension, it shows a gradually increasing trend.

The second step is to reduce the error in the process of path planning and optimal scheme formulation and improve the guidance efficiency of ice and snow movement trajectory and path analysis. In this process, we need to use the discriminant function to judge the planning efficiency. The discriminant function *Q*(*s*) before optimization is

(3) $$\begin{array}{c} Q\left(s\right)=\frac{\sqrt{3s^{3}+3s^{2}+4s+1}}{s}. \end{array}$$

After adding anti-interference factor *e*, the optimized discriminant function *Q* ′(*s*) is

(4) $$\begin{array}{c} Q^{\prime }\left(s\right)=\frac{\sqrt{5s^{3}+5s^{2}+3s+1}/3s+1}{e+3}, \end{array}$$

*s* is the trajectory data of ice and snow movement; *e* is the anti-interference factor.

In the third step, according to the difference of position dynamic stability of different types of ice and snow sports, the position of athletes can be updated dynamically:

(5) $$\begin{array}{c} T\left(s\right)=\frac{7s^{3}+7s^{2}+5s+3}{s+5s^{-1}}. \end{array}$$

The location function with dynamic update strategy is

(6) $$\begin{array}{c} T{\;}^{\prime }\left(s\right)=\frac{\sqrt{7s^{3}+7s^{2}+5s+3/s+5s^{-1}}}{r^{s}+s+s^{-1}}, \end{array}$$

*s* is the trajectory data of ice and snow movement; *r* is the dynamic change factor. In this way, after several interactive cycles of two-way gait information, the best strategy data will be obtained according to the data analysis method, and the specific path trajectory information in line with the lowest normal ice and snow movement trajectory will be generated; that is, the data vector value of the normal boundary of an ice and snow movement path position signal and the longitude and latitude coordinates of the known position information will be compared and analyzed. In this way, the information analysis and recording of ice and snow movement track, path scheme, and coordinate longitude and latitude can be realized under the condition of “MNN algorithm.” The simulation results are shown in Figure 4. As can be seen from Figure 4, with the increase of simulation times, the corresponding coincidence index of ice and snow movement trajectory (according to the commonly used empirical value, the maximum value of coincidence is 2.85) shows a gradually increasing trend, which is also in line with the law of ice and snow movement in path planning.

In MNN algorithm, the longitude and latitude analysis function *P*(*s*) and trajectory analysis function *H*(*s*) are

(7) $$\begin{array}{c} P\left(s\right)=\frac{9s^{3}+7s^{2}+s^{x}+5}{3s^{x}+5s^{-1}+1},\\ H\left(s\right)=\frac{7s^{x+1}+7s^{x}+7s^{x-1}+9}{3s^{x}+5s^{x-1}+3}. \end{array}$$

*s* is the track data of ice and snow movement and *x* is the longitude and latitude information. The ice and snow movement path planning mode based on the longitude and latitude coordinate information of the path can also realize the self storage and cloud computing functions of the data information generated in this process. Therefore, the more the accumulated historical data of ice and snow movement trajectory and path location information, the stronger the self-learning ability and intelligent planning guidance scheme of the system. This adaptive path planning and tracking method can complete the intelligent path planning and error rate control of ice and snow movement with high accuracy. The analytic simulation results of this ice and snow movement path planning model for two different target path planning schemes are shown in Figure 5. According to the simulation results in Figure 5, it can be seen that, with the control of the error rate, the intelligent degree of the path planning solution, whether it is time first or distance first, tends to rise first and then fall. Therefore, it can be considered that the path planning solution has little effect on time or distance.

### 3.3. Different Ice and Snow Sports Path Planning Guidance Scheme and Optimization Improvement Strategy

In the process of reconstructing the trajectory of ice and snow, because different object will produce different deviations in the process of space motion, especially in the real-time dynamic position signal processing of balls, we use MNN algorithm with adaptive characteristics. In order to improve the effect of different ice and snow movement path planning by MNN algorithm, it is necessary to optimize the MNN algorithm, and the optimization process is realized by the partial local method. In the process of distribution, the threshold value *E* is selected according to the following criteria:

(8) $$\begin{array}{c} r\left(s\right)=\frac{1}{\sqrt{5s^{t}+5s^{t-1}+3s}},\\ e\left(s\right)=\frac{r}{\sqrt{5s^{t+r}+5s^{t-r}+3s^{r}}},\\ E=\frac{e+r}{e^{t+r}+e^{t-r}+e^{r}}. \end{array}$$

*s* is the trajectory data of ice and snow movement, *t* is the eigenvalue information, *r*(*s*) is the result of the first distribution, and *e*(*s*) is the result of the multiple distribution.

In the process of tracking and reconstructing the track of ice and snow movement, MNN algorithm needs to select its motion feature in the process of spatial motion analysis for probability state, that is, the selection of ice and snow motion feature factor based on the whole crowd target, and then detect and analyze according to different path feature functions, whose path feature function *M*(*s*) is

(9) $$\begin{array}{c} M\left(s\right)=\frac{\sqrt[{3}]{3s^{t+1}+3s^{t}+2s^{t-1}+8}}{\sqrt{5s^{t}+5s^{t-1}+8}}. \end{array}$$

After adding the tracking condition, the path characteristic function *M* ′(*s*) is

(10) $$\begin{array}{c} M{\;}^{\prime }\left(s\right)=\frac{t+s^{2}}{t-s}+\frac{\sqrt[{3}]{3s^{t+1}+3s^{t}+2s^{t-1}+8}}{\sqrt{5s^{t}+5s^{t-1}+8}}, \end{array}$$

where *s* is the track data of ice and snow movement and *t* is the eigenvalue information. In the aspect of path planning for ice and snow sports, this model will use the existing ice and snow sports big data and the path planning information database stored in the cloud, combined with the data analysis factor, to analyze the adaptive disturbance of the limit weight value obtained from the optimized MNN algorithm, and then use the MNN algorithm to subdivide specific ice and snow sports information. According to the differences of different types of ice and snow movement paths, the integrity of them is sorted, and then the sorting results are discretized according to different weight indexes, and the path factors related to the optimization strategy are marked, and the marking results are transmitted to the optimal path planning scheme database. The expressions of the standard function *B*(*s*) and the discrete weight solving function *J*(*s*) of the optimal path planning scheme are as follows:

(11) $$\begin{array}{c} B\left(s\right)=\frac{t^{2s}+s^{2t}}{t^{s}-s^{t}},\\ J\left(s\right)=\frac{t^{2s}-s^{2t}}{\sqrt{t^{s}+s^{t}}}+\frac{B^{t}\left(s\right)+tB\left(s\right)}{B^{2t}\left(s\right)-tB\left(s\right)}, \end{array}$$

where *s* is the track data of ice and snow movement and *t* is the eigenvalue information. The simulation results of path selection and the number of scattered points are shown in Figure 6.

As can be seen from Figure 6, with the increase of the number of key points of the path, the scattered points of the path in the four different schemes also show different changing rules with obvious characteristics. This is because MNN algorithm first selects the data coding for the ice and snow trajectory and then classifies the different types of parameter data groups. Then the MNN algorithm is used to solve the local optimization of the processed path database, and the internal change law is analyzed. In order to realize the optimization of the path selection process, we will form the vector matrix group with key characteristics from the path parameters and other information generated in the process of ice and snow movement and input it into the path planning guidance model. These vector groups produce different vector eigenvalues according to the different path trajectories of ice and snow movement. Therefore, the spatial position of the original ice and snow movement in the process of path selection is analyzed by using the transformed matrix sequence.

## 4. Result Analysis and Discussion

### 4.1. Experimental Process of Ice and Snow Path Planning Guidance Model Based on MNN Algorithm

Before the beginning of the experiment, we set up a model of ice and snow trajectory reconstruction and path planning based on the characteristic parameters and path differences. The model centers on the dynamic movement process of ice and snow athletes and takes the differences of different ice and snow trajectories and different path schemes as the core evaluation index. The reconstruction effect and path planning strategy of ice and snow trajectory are evaluated. The experimental process is shown in Figure 7.

As can be seen from Figure 7, with the increase of the number of dynamic signals (the number of experiments), the completion degree of path planning gradually increases until it becomes stable. This is because the more the number of signals, the more the amount of calculation required, and so the higher the degree of coincidence. Moreover, the MNN algorithm has better reliability and data stability. Compared with other methods, it also has better scientific reference in the error control of the optimal solution of the path. This is because in the ice and snow movement path planning model, different ice and snow movement trajectories, and path data are taken as the experimental objects. Through the tracking process of different ice and snow movement tracks, the intelligence and convenience of ice and snow movement path planning scheme are evaluated. It is mainly based on the automatic analysis strategy and multidata comparison method of conventional ice and snow sports path planning at the big data level. Then, through the detection and quantitative processing of the motion data in ice and snow movement, the analysis of different types of ice and snow movement trajectories and the planning and feasibility prediction of the optimal path are realized. On this basis, with the help of the idea of nearest neighbor strategy, the optimal path planning guidance for different types of ice and snow sports is realized and displayed by three-dimensional visualization method. This is also an innovation of the intelligent analysis model based on MNN algorithm in the research of real-time path planning and intelligent data processing methods of ice and snow sports.

### 4.2. Analysis of Experimental Results

The stability test results of the experimental results of snow and ice trajectory reconstruction based on MNN algorithm and other path planning methods are shown in Figure 8, and the evaluation results of the snow and ice path planning guidance model based on MNN algorithm and other path planning methods are shown in Figure 9.

It can be seen from Figures 8 and 9 that, with the increase of the number of experiments, the stability of the overall path planning is significantly improved. This is because, with the increase of the number of experiments, certain error data will be eliminated in each calculation process (which can be judged according to the coincidence degree) and in the process of analyzing the experimental results. We find that, in the process of feature extraction, the reconstruction of ice and snow trajectory is based on the data stored in the hardware of traditional detection equipment, and the detection process is mainly direct contact detection, while the noncontact real-time motion space signal detection is rare. Therefore, in the detection of ice and snow movement, a standard evaluation model of ice and snow movement trajectory data is determined in advance (in order to determine the key detection nodes). Therefore, this paper studies the processing object based on the spatial position change of the ball randomly selected from the local ice and snow movement set of multiple targets to be detected. By comparing and analyzing the real-time analysis model of the ball's spatial position and the big data system of sports ice and snow trajectory, it is easy to know that, in the process of the change of the two ball's spatial position, if there is a high degree of structural similarity in the group, the numerical difference of the ice and snow trajectory between them is very small. This shows that the accuracy of this model is very high.

Finally, this study takes two similar ice and snow movement path schemes in sports as a group of tracking research objects, and a random ice and snow movement path as the control object. One of the groups is that the ice and snow movement path is known (the ice and snow movement path and other information are known). The other group is that the track of ice and snow movement is unknown (the initial track and path of ice and snow movement are known, but the details of the specific motion path are unknown). It is found that there is a high similarity in the process of reconstructing the ice and snow trajectory in the two kinds of data, and the error is 1.2% and 2.3%, respectively. In the guidance scheme of ice and snow path planning based on MNN algorithm, the intelligent path planning scheme given by MNN algorithm is in good agreement with the real optimal path planning scheme. Therefore, the research results of this experiment show that the ice and snow movement path planning model based on MNN algorithm combined with the characteristics of ice and snow movement and data reliability, intelligent planning for different types of ice and snow movement path planning scheme, and its high degree of coincidence, in line with the actual application needs. Therefore, the experimental results show that the ice snow path planning method based on MNN algorithm can be applied to the dynamic analysis of ice snow trajectory and the guidance of the optimal path allocation after the game.

## 5. Conclusion

In recent years, there are many problems in the research of ice and snow sports, such as the inefficient path planning of ice and snow sports, less application scope, and so on. Therefore, the reform of traditional ice and snow sports path planning method is more and more urgent. Based on this, this paper studies the path planning model of ice and snow sports based on MNN algorithm and designs the dynamic tracking method of intelligent path planning of ice and snow sports based on the three-dimensional trajectory model. Through the research of three aspects in the process of ice and snow movement, the ice and snow movement path planning guidance system based on the minimization strategy is constructed. Finally, the MNN algorithm and the optimized iterative data analysis model are used to analyze the characteristics of the screening results and the intelligent path planning process. The experimental results show that the model can make full use of the intelligent path planning strategies of different types of ice and snow sports, achieve the integrity of the intelligent path of ice and snow sports, efficiently carry out the customized analysis of the factors affecting the ice and snow sports path planning, and improve the efficiency of path planning. However, this paper only focuses on the path planning method of ice and snow movement and does not take the directional capture efficiency and the potential impact of error into account. Therefore, the ice and snow movement path planning model has some room for improvement.

## Figures and Tables

**Figure 1:** Data processing process under the MNN algorithm.

**Figure 2:** Processing process of ice and snow movement path planning guidance system.

**Figure 3:** Simulation analysis results of different ice and snow sports data.

**Figure 4:** The coincidence index of ice and snow trajectory under different simulation times.

**Figure 5:** Analytical simulation results of path planning schemes for two different goals.

**Figure 6:** Reconstruction model of volleyball sports track based on filtering algorithm.

**Figure 7:** Experimental process of intelligent planning of ice and snow sports path.

**Figure 8:** Stability of experimental results under different experimental times.

**Figure 9:** Evaluation results of different guidance models for path planning of ice and snow sports.

## Data Availability

The experimental data used to support the findings of this study are available from the corresponding author upon request.

## References

[1] Zhang Z., Park C. Y., Theesfeld C. L., Troyanskaya O. G. (2021). An automated framework for efficiently designing deep convolutional neural networks in genomics. *Nature Machine Intelligence*.

[2] Hewamalage H., Bergmeir C., Bandara K. (2021). Recurrent neural networks for time series forecasting: Current status and future directions. *International Journal of Forecasting*.

[3] Dewangan D. K., Sahu S. P. (2021). RCNet: road classification convolutional neural networks for intelligent vehicle system. *Intelligent Service Robotics*.

[4] Elnaz P., Elham P., Nizamettin A. (2018). Gene selection using hybrid binary black hole algorithm and modified binary particle swarm optimization. *Genomics*.

[5] Zenke F., Vogels T. P. (2021). The remarkable robustness of surrogate gradient learning for instilling complex function in spiking neural networks. *Neural Computation*.

[6] Zhang A., Xiang Z., Jin T. (2018). Exploring influence of different gait trajectories on major muscle fatigue of a lower human limb. *Mechanical Science & Technology for Aerospace Engineering*.

[7] Thieberger P., Gassner D., Hulsart R. (2018). Fast readout algorithm for cylindrical beam position monitors providing good accuracy for particle bunches with large offsets. *Review of Scientific Instruments*.

[8] Wang J., Yang Y., Wang T., Sherratt R. S., Zhang J. (2020). Big data service architecture: a survey. *Journal of Internet Technology*.

[9] Qi C.-C. (2020). Big data management in the mining industry. *International Journal of Minerals, Metallurgy and Materials*.

[10] Bragazzi N. L., Dai H., Damiani G., Behzadifar M., Martini M., Wu J. (2020). How big data and artificial intelligence can help better manage the COVID-19 pandemic. *International Journal of Environmental Research and Public Health*.

[11] Fischer C., Pardos Z. A., Baker R. S. (2020). Mining big data in education: affordances and challenges. *Review of Research in Education*.

[12] Guo K., Xu F., Wang Y., Liu Y., Dai Q. (2018). Robust non-rigid motion tracking and surface reconstruction using $L_0$ regularization. *IEEE Transactions on Visualization and Computer Graphics*.

[13] Xia J., Wang J., Niu S. (2020). Research challenges and opportunities for using big data in global change biology. *Global Change Biology*.

[14] Grattarola D., Alippi C. (2021). Graph neural networks in TensorFlow and keras with spektral [application notes]. *IEEE Computational Intelligence Magazine*.

[15] Miles C., Bohrdt A., Wu R. (2021). Correlator convolutional neural networks as an interpretable architecture for image-like quantum matter data. *Nature Communications*.

[16] Janson L., Ichter B., Pavone M. (2018). Deterministic sampling-based motion planning: Optimality, complexity, and performance. *The International Journal of Robotics Research*.

[17] Saeed J., Zeebaree S. (2021). Skin lesion classification based on deep convolutional neural networks architectures. *Journal of Applied Science and Technology Trends*.

[18] Singh Y., Sharma S., Sutton R., Hatton D., Khan A. (2018). A constrained A*∗* approach towards optimal path planning for an unmanned surface vehicle in a maritime environment containing dynamic obstacles and ocean currents. *Ocean Engineering*.

[19] Wu Y. (2019). Coordinated path planning for an unmanned aerial-aquatic vehicle (UAAV) and an autonomous underwater vehicle (AUV) in an underwater target strike mission. *Ocean Engineering*.

[20] Khanra S., Dhir A., Mäntymäki M. (2020). Big data analytics and enterprises: a bibliometric synthesis of the literature. *Enterprise Information Systems*.

[21] Hamilton R. H., Sodeman W. A. (2020). The questions we ask: Opportunities and challenges for using big data analytics to strategically manage human capital resources. *Business Horizons*.

[22] An N., Qi Yan W. (2021). Multitarget tracking using Siamese neural networks. *ACM Transactions on Multimedia Computing, Communications, and Applications*.

[23] Sun H., Xu M. T., Wang X. Q. (2018). Comparison thigh skeletal muscles between snowboarding halfpipe athletes and healthy volunteers using quantitative multi-parameter magnetic resonance imaging at rest. *Chinese Medical Journal*.

[24] Halverson J., Maiti A., Stoner K. (2021). Neural networks and quantum field theory. *Machine Learning: Science and Technology*.

[25] Çolak A. B. (2021). An experimental study on the comparative analysis of the effect of the number of data on the error rates of artificial neural networks. *International Journal of Energy Research*.

[26] Thanh P. D., Binh H. T. T., Trung T. B. (2020). An efficient strategy for using multifactorial optimization to solve the clustered shortest path tree problem. *Applied Intelligence*.

